# Determining the appropriate level of farmyard manure biochar application in saline soils for three selected farm tree species

This article has been retracted.

**DOI:** 10.1371/journal.pone.0265005

**Published:** 2022-04-06

**Authors:** Muhammad Talha Bin Yousaf, Muhammad Farrakh Nawaz, Ghulam Yasin, Hefa Cheng, Irfan Ahmed, Sadaf Gul, Muhammad Rizwan, Abdur Rehim, Qi Xuebin, Shafeeq Ur Rahman

**Affiliations:** 1 Department of Forestry and Range Management, University of Agriculture, Faisalabad, Pakistan; 2 Department of Forestry, Range and Wildlife Management, The Islamia University Bahawalpur, Bahawalpur, Pakistan; 3 Department of Forestry and Range Management, Bahauddin Zakariya University Multan, Multan, Pakistan; 4 MOE Laboratory for Earth Surface Processes, College of Urban and Environmental Sciences, Peking University, Beijing, China; 5 Department of Botany, University of Karachi, Karachi, Pakistan; 6 Department of Environmental Sciences and Engineering, Government College University, Faisalabad, Pakistan; 7 College of Agriculture, Department of Soil Science, Bahadur Sub-Campus Layyah, Bahauddin Zakariya University, Multan, Pakistan; 8 Farmland Irrigation Research Institute, Chinese Academy of Agricultural Sciences, Xinxiang, China; 9 School of Environment and Civil Engineering, Dongguan University of Technology, Dongguan, China; Government College University Faisalabad, Pakistan, PAKISTAN

## Abstract

Salinity is a global problem, and almost more than 20% of the total cultivated area of the world is affected by salt stress. Phytoremediation is one of the most suitable practices to combat salinity and recently biochar has showed the tremendous potential to alleviate salt-affected soils and enhance vegetation. Trees improve the soil characteristics by facilitating the leaching of salts and releasing organic acids in soil. Moreover, in the presence of trees, higher transpiration rates and lower evaporation rates are also helpful in ameliorating salt affected soils. This study was designed to check the effect of different levels of biochar on the morph-physiological characteristics of three important agroforestry tree species: *Eucalyptus camaldulensis*, *Vachellia nilotica*, *and Dalbergia sissoo*, in saline soils. Farmyard manure biochar was applied at the rate of 3% (w/w), 6% (w/w), and 9% (w/w) to find appropriate levels of biochar for promoting the early-stage trees growth under saline conditions. Results of the current study revealed that maximum shoot length (104.77 cm), shoot dry weight (23.72 g), leaves dry weight (28.23 g), plant diameter (12.32 mm), root length (20.89 cm), root dry weight (18.90 g), photosynthetic rate (25.33 μ moles CO_2_ m^-2^s^-1^) and stomatal conductance (0.12 mol H_2_O m^-2^ s^-1^) were discovered in the plants of *Eucalyptus camaldulensis* at the rate of 6% (w/w). All tree species showed better results for growth and physiological characteristics when biochar was applied at the rate of 6% (w/w). In comparison, a decreasing trend in growth parameters was found in the excessive amount of biochar when the application rate was increased from 6% (w/w) to 9% (w/w) for all three species. So, applying an appropriate level of biochar is important for boosting plant growth in saline soils. Among different tree species, *Vachellia nilotica* and *Eucalyptus camaldulensis* both showed very promising results to remediate salt affected soils with *Vachellia nilotica* showing maximum potential to absorb sodium ions.

## 1. Introduction

Soil is one of the most important constituents of the natural ecosystem. Soil acts as a junction among different important environmental entities like earth, air and water [1, 2]. Problematic soils can be defined as soils having feeble physical, chemical, and biological characteristics, which can inhibit plant growth [3]. Salt affected soils have high concentrations of dissolved salts and or/ high levels of adsorbed sodium in the soil matrix. If the soils have the values of EC above than 4 dS m^−1^ and values of SAR or ESP below 13 or 15, respectively, the soils are referred to as saline soil. Some studies suggested that almost 20% of the total cultivated land of the world and over 10% of the total irrigated land is disturbed by salinity [4–6]. Some countries are affected with salts to such an extent that 50% of total cultivated land is not cultivable due to salinity [7, 8]. In Pakistan, 4.5 million hectares (Mha) out of total cultivable land (21 Mha) is affected by salinity and waterlogging [9]. Therefore, to ensure a continuous food supply, soil salinity should be addressed on a priority basis to avoid food scarcity and hunger risks [10].

Soil salinity severely affects soil health and soil fertility. Plants grown in saline soils face a lot of problems like nutrients imbalance, ion toxicity, and oxidative stress [11–13]. Many methods are used to reclaim salt-affected soils, including physical, chemical, biological, and combination of different techniques [14, 15]. Phytoremediation is a clean, proficient, economical and environment-friendly technique to remove toxic pollutants by using green plants [16, 17]. Forestry and agroforestry are the best-suited options to make these degraded soils productive, and multipurpose trees on these soils have numerous benefits [18–20].

Biochar is one of the most important organic amendments produced by partial burning of materials or biomass rich in carbon contents such as agricultural residues [21]. Biochar has gained significant importance in recent times, and it is reported that biochar has numerous benefits like soil fertility enhancement, the potential to sequester carbon, the capability of immobilizing pollutants of organic and inorganic nature [22, 23]. Application of biochar under abiotic stresses like salt and drought stress can enhance the growth of plants, increase yield, and improve biomass and nutrient uptake in plants [24–26]. Biochar has also shown very positive results in improving soil physicochemical properties [26–28].

It is estimated that almost 1.4 billion cows are present in the world. These cows produce nearly 4.2 million dung per year as waste material [29]. Different types of techniques are used to solve their disposal problem. Traditionally this material is used to form fertilizer through composting or as a fuel for biogas production [30, 31]. The conversion of dung into biochar has gained significant importance in recent times. Proteins, cellulose, hemicelluloses, and other essential nutrients are present in huge quantities in cow dung [29, 32]. So, dung can have proved to be a vital source for the production of biochar. Farmyard manure biochar (FYMB) is reported to enhance the crop yield and Physico-chemical properties of soils [33]. It can adsorb perchlorate from water [34] and helpful in combating heavy metal stress in perennial woody vegetation [35]. Among different types of biochar, farmyard manure biochar showed very promising results in enhancing the growth of agroforestry tree species [36]

It is important to find the optimum level of FYMB for afforestation of saline soils. In this pioneering study, the three most important agroforestry tree species were used: *Vachellia nilotica*, *Dalbergia sissoo and Eucalyptus camaldulensis*.

*Vachellia nilotica* is a valuable member of the plant family *Fabaceae*, having the potential to tolerate salinity [37–40]. *Dalbergia sissoo* is one of the most important and preferred leguminous agroforestry tree species grown in Pakistan, India, and Nepal [41]. *D*. *sissoo* has been used to ameliorate sodic soils [42]. The *Eucalyptus* genus is considered to be one of the most important trees for industrial plantations. It is native to the Australian continent, and it’s neighboring countries (Tran et al. 2018; Yang et al. 2018). *Eucalyptus* covers almost 10,000 ha land in Pakistan, and it is a part of almost every major afforestation program in the country [43, 44].

This study was designed to check the phytoremediation potential of three selected agroforestry species (*V*. *nilotica*, *D*. *sissoo*, *and E*. *camaldulensis*) and the effect of different levels of farmyard manure biochar on the growth of these species and finding the appropriate level of biochar to reclaim salt degraded soil through afforestation.

## 2. Materials and methods

A pot experiment was conducted in the nursery area of the Department of Forestry and Range Management (FRM), University of Agriculture Faisalabad (UAF) (31° 25’57" N, 73° 04’ 21" E) from March 2017 to August 2017. Climatic conditions during the pot experiment were collected from Agricultural Metrology Cell, UAF, and described in Table 1.

**Table 1:** Climatic conditions data during the year 2017.

Month	Average Max. Temp. (°C)	Average Min. Temp. (°C)	Precipitation (mm)	Sunshine Duration (Hours)	ET₀(mm)
**January**	17.6	08.2	11.5	03.6	00.9
**February**	23.3	10.2	4.1	06.6	01.9
**March**	27.3	14.2	16.2	07.2	02.7
**April**	37.7	20.9	28.3	09.2	05.2
**May**	41.1	26.0	10.1	10.4	05.7
**June**	39.8	27.3	41.6	09.38	05.3
**July**	38.5	28.9	117.2	07.0	04.0
**August**	38.1	28.6	66	07.9	03.8

### 2.1. Characteristics of Salt affected soil

A comprehensive survey of sat affected soils was carried out in district Faisalabad, Pakistan. Random samples were collected from different sites with the help of an auger. After collection, the Electrical conductivity (EC) and pH of all soil samples were determined. The site with poor soil conditions and high EC was selected for the current study. Soil was naturally affected by salt stress as it can be seen by it’s properties in Table 2. Detailed soil analysis was performed to examine various physicochemical characteristics of soil according to the US Salinity Laboratory Staff [45]. Before the initiation of the experiment, physicochemical characteristics of soil are given in Table 2.

**Table 2:** Physicochemical characteristics of the soil before the initiation of the experiment.

Textural class	Sandy Loam
Sand (%)	60 ± 1
Silt (%)	25 ± 0.5
Clay (%)	15 ± 0.3
Saturation (%)	28 ± 1
pH	8.5 ± 0.3
EC (dS/m)	20.5 ± 9
TSS (mmol/L)	205 ± 20
CO_3_^2-^ (mmol/L)	10 ± 2
HCO_3_^-^ (mmol/L)	30 ± 4
Cl^-^ (mmol/L)	140 ± 19
Ca^2+^ + Mg^2+^ (mmol/L)	12 ± 4.5
Na^+^ (mmol/L)	160 ± 15.2
K^+^ (mmol/L)	47 ± 7
OM (%)	0.64 ± 0.03

### 2.2. Preparation of biochar and it’s characteristics

Farmyard manure biochar was selected because it produced best results among different types of biochar against salinity [36]. Raw material for preparing biochar was collected from the farm area of the Agronomy field UAF. Biochar was prepared by slow pyrolysis of dung cakes for 3 hours durations. Batch pyrolysis temperature-controlled unit was used to produce biochar at 450°C. The pyrolysis conditions are described earlier by [46].Biochar was prepared in Agro-climatology lab of UAF and the characteristics of biochar are given in Table 3.

**Table 3:** Physicochemical characteristics of Farmyard Manure Biochar.

pH	7.0
EC (dS/m)	2.08
TSS (mg/kg)	20.8
CO_3_^2-^(mg/kg)	(-)
HCO_3_^-^(mg/kg)	8
Cl^-^ (mg/kg)	4
Ca^2+^ + Mg^2+^ (mg/kg)	13.2
Na^+^ (mg/kg)	3.4
K^+^(mg/kg)	7.2
OM (%)	95.4
TOC (%)	70.2

### 2.3. Planting material and application rates of biochar

Three agroforestry tree species (*Eucalyptus camaldulensis*, *Vachellia nilotica*, *and Dalbergia sissoo*) were selected for this study. Uniform-sized disease-free seedlings of these species were collected from the arboretum of the nursery of the Department of Forestry and Range Management and were grown in pots. The internal diameter and height of the pots were 10 inches. 10 kg of soil was present in one pot. Biochar was applied at three different rates 3% (w/w), 6% (w/w), and 9% (w/w). So, there were four treatments, including control and three species. For every treatment, there were three replications, and for each replication, 3 plants were grown. So, there were nine plants for every treatment. Groundwater was used to irrigate the plants, and the characteristics of the water used for this experiment are given in Table 4.

**Table 4:** Characteristics of tap water of nursery.

pH	7.29
EC (dS/m)	0.669
TSS (mg/L)	6.699
Carbonates	(-)
Bi Carbonates (mg/L)	4.8
Ca + Mg (mg/L)	3
Chlorides (mg/L)	2.5
RSC	1.8
Sodium (mg/L)	0.69

### 2.4. Harvesting of plants

Plants were harvested after six months. At the time of harvesting, the growth parameters and physiological characteristics of plants were measured. Moreover, sodium and potassium contents in different plant parts were also measured. In addition to that post-harvest physicochemical characteristics of soil were also determined.

#### 2.4.1. Growth and physiological attributes

Shoot length and root length were measured with the help of measuring tape. Collar diameter(mm) of shoots of the three selected species were measured with the help of a digital Vernier caliper. Dry weight (g) of roots, shoots, branches, and leaves was taken by drying them in an oven (101-1AB) at 75˚C till the constant weight was obtained. Photosynthetic rate (μ mol of CO_2_ m^-2^ s^-1^) transpiration rate (mmol O_2_ m^-2^ s^-1^), stomatal conductance (mmol H_2_O m^-2^ s^-1^), and sub-stomatal CO_2_ concentration (μ mol of CO_2_ mol^-1^ air) were measured on the second upper fully expanded leaves, using a system LCA-4 ADC portable infrared gas analyzer (Analytical Development Company, Hoddesdon, England). Chlorophyll measured in SPAD values was also performed on the third upper leaves using a chlorophyll meter (SPAD-502, Konika Minolta Sensing Inc., Japan).

#### 2.4.2. Ionic contents

At the time of harvesting, digestion of the plant samples was performed according to the procedures described earlier [47]. After digestion, the mixture was cooled to room temperature, diluted to 25 ml with distilled water, and stored in an air-tight bottle for ionic analysis. The ionic concentration for Na^+^ and K^+^ in plant samples was determined by Jenway PFP-7 flame photometer with the help of standard solutions using reagent grade salt of NaCl and KCl, respectively according to the protocols described earlier [45, 48].

### 2.5. Statistical analysis

The data was analyzed by using factorial under CRD using computer-based software IBM SPSS 25.0 for windows. Tukey HSD was also applied to differentiate any significant differences between treatments.

## 3. Results

### 3.1. Growth attributes

Results of different growth parameters against four different treatments are depicted in Fig 1. Shoot length, root length, shoot diameter, shoot dry weight, root dry weight, dry leaf weight, and dry branch weight was measured. This study indicated that almost all the growth parameters showed better results when treated with farmyard manure biochar (FYMB) compared to control. Maximum growth was found in the plants treated with 6% biochar, whereas control treatment plants showed minimum growth for all three selected agroforestry tree species. Shoot length, root length, and shoot diameter for all the species against all the treatments were found in the range of 48.89–104.78 cm, 8.33–20.89 cm, and 3.68–12.42 mm, respectively. A dry weight of shoot, root, leaf, and branches were found in the range of 9.32–23.24 g, 9.03–18.90 g, 8.06–28.20 g, 5.97–28.49 g, respectively. The general trend of species against all treatments for the shoot, root, and leaf dry weight was recorded as *E*. *camaldulensis > V*. *nilotica > D*. *sissoo*, whereas branch dry weight trend was found to be as *V*. *nilotica > E*. *camaldulensis > D*. *sissoo*. Order for treatments for growth parameters is FYMB 6% > FYMB 9% > FYMB 3% > Control. All treatments of biochar showed better results as compared to control. FYMB 6% was found to be best among all treatments.

**Fig 1:** Growth parameters of plants against three different levels of Farmyard Manure Biochar. These values are three replicates, and for each replication, there were three plants (n = 9). The difference between lower case letters indicates that values are significantly (p < 0.05) different from each other.

### 3.2. Physiological parameters

Results of different physiological parameters of three selected agroforestry species against different levels of farmyard manure biochar are depicted in Fig 2. Chlorophyll contents, photosynthetic rate, stomatal conductance, transpiration rate and sub-stomatal CO_2_ concentration were found in the range of 34.14–65.22 (SPAD values), 7.10–25.33 (μ moles CO_2_ m^-2^ s^-1^), 0.02–0.12 (mol H_2_Om^-2^ s^-1^), 1.62–1.52 (mmol O_2_ m^-2^ s^-1^) and 179.44–318.33 (μ moles CO_2_ mol^-1^ air) respectively. *Eucalyptus camaldulensis* showed the best physiological attributes among all three species, whereas *Dalbergia sissoo* showed minimum physiological attributes against all treatments. The general trend of species against all treatments for physiological attributes was recorded as *E*. *camaldulensis > V*. *nilotica > D*. *sissoo*. Farmyard manure biochar applied at the rate of 6% was found to be best among all treatments. Order for treatments for physiological attributes is FYMB 6% > FYMB 9% > FYMB 3% > Control. The application of biochar showed promising results in improving the physiological attributes of plants grown in salt-affected soils.

**Fig 2:** Physiological attributes of plants against three different levels of Farmyard Manure Biochar. These values are the means of three replicates, and for each replication, there were three plants (n = 9). The difference between lower case letters indicates that values are significantly (p < 0.05) different from each other.

### 3.3. Ionic parameters

Trees have excellent potential to remediate saline soils through phytoremediation. Results of this study revealed that different treatments showed significantly different results as compared to control. The concentration of sodium, potassium, and chlorides in roots and shoots of all three selected agroforestry species are given in Fig 3. Maximum shoot sodium (5.82 mg/g DW) and shoot chlorides (8.80 mg/g DW) were found in the plants of untreated *Vacellia nilotica*. Maximum shoot potassium was found in plants of *Eucalyptus camaldulensis* treated with FYMB 6% (6.03 mg/g DW), slightly higher than FYMB 9% (5.28 mg/g DW). Maximum root sodium (7.81 mg/g DW) and chlorides (10.56 mg/g DW) were found in the plants of *Vachellia nilotica* under control treatment, whereas maximum root potassium was found in the plants of *Eucalyptus camaldulensis* treated with FYMB 9% (5.40 mg/g DW) slightly above than the plants treated with FYMB 6% (5.33 mg/g DW) and minimum root potassium (0.67 mg/g DW) was present in the untreated plants of *Dalbergia sissoo*. Biochar increased potassium and reduced sodium, especially in the root zone of plants.

**Fig 3:** Ionic contents of plants against three different levels of Farmyard Manure Biochar. These values are means of three replicates, and for each replication, there were three plants (n = 9). The difference between lower case letters indicates that values are significantly (p < 0.05) different from each other.

### 3.4. Post-harvest soil characteristics

Post-harvest soil characteristics are given in Table 5. pH of the soil was reduced for all the treatments from the initial pH of the soil, but minimum pH was found in the plants of control treatment. By applying biochar, electrical conductivity was reduced for all the treatments. Minimum EC along with TSS and SAR was showed by the plants of *Eucalyptus camaldulensis* treated with FYMB 6%, whereas untreated plants of Dalbergia sissoo showed maximum. Organic matter and saturation (%) were also increased using organic amendments, with FYMB 9% giving the best results. The trend of treatments for improving soil characteristics was FYMB 6% > FYMB 9% > FYMB 3% > Control. Among species, *E*. *camaldulensis* was found to be best for reclamation of soil, and *D*. *sissoo* was found to be least effective. Data regarding different soil characteristics are given in Table 5.

**Table 5:** Effect of different levels of biochar and selected agroforestry trees species on post-harvest soil characteristics.

	Control			FYMB 3%			FYMB 6%			FYMB 9%		
	Sp. 1	Sp. 2	Sp. 3	Sp. 1	Sp. 2	Sp. 3	Sp. 1	Sp. 2	Sp. 3	Sp. 1	Sp. 2	Sp. 3
**pH**	7.73a ± 0.08	7.77a ± 0.08	7.77a ± 0.08	8.07abc ± 0.08	8.20a ± 0.08	8.20a ± 0.08	7.93abc ± 0.08	7.93abc ± 0.08	8.00abc ± 0.08	7.97abc ± 0.08	8.10ab ± 0.08	8.10ab ± 0.08
**EC (dS/m)**	8.29b ± 0.28	8.71b ± 0.28	12.41a ± 0.28	3.77ef ± 0.28	4.41de ± 0.28	6.71c ± 0.28	3.22f ± 0.28	3.22f ± 0.28	5.19d ± 0.28	4.65de ± 0.28	5.23d ± 0.28	6.98c ± 0.28
**TSS(mmol/L)**	82.90b ± 2.82	87.10b ± 2.82	124.10a ± 2.82	37.70ef ± 2.82	44.10de ± 2.82	67.07c ± 2.82	32.17f ± 2.82	32.17f ± 2.82	51.93d ± 2.82	46.47de ± 2.82	52.27d ± 2.82	69.80c ± 2.82
CO_3_^2-^(mmol/L)	(-)	(-)	(-)	(-)	(-)	(-)	(-)	(-)	(-)	(-)	(-)	(-)
HCO_3_^-^(mmol/L)	3.20cd ± 0.22	4.44ab ± 0.22	4.51a ± 0.22	5.44c ± 0.22	5.97bc ± 0.22	6.18abc ± 0.22	3.65e ± 0.22	3.65e ± 0.22	3.83de ± 0.22	4.11de ± 0.22	4.22de ± 0.22	4.53d ± 0.22
Cl^-^ (mmol /L)	40.00c ± 1.1	51.00b ± 1.1	60.00a ± 1.1	18.00g ± 1.1	20.00g ± 1.1	25.00ef ± 1.1	14.00h ± 1.1	14.00h ± 1.1	26.67ef ± 1.1	25.00ef ± 1.1	28.00de ± 1.1	30.63d ± 1.1
Ca^2+^+Mg^2+^ (mmol/L)	3.73b ± 0.7	3.73b ± 0.7	3.83b ± 0.7	6.77ab ± 0.7	7.20a ± 0.7	7.20a ± 0.7	7.93a ± 0.7	7.93a ± 0.7	7.87a ± 0.7	8.47a ± 0.7	9.20a ± 0.7	9.14a ± 0.7
Na^+^ (mmol/L)	48.00b ± 1.23	51.00b ± 1.23	62.33a ± 1.23	21.33def ± 1.23	23.00de ± 1.23	30.00c ± 1.23	17.00f ± 1.23	17.00f ± 1.23	23.33de ± 1.23	19.67ef ± 1.23	21.33def ± 1.23	25.67cd ± 1.23
**SAR**	35.23b ± 1.69	37.41b ± 1.69	45.50a ± 1.69	11.78bc ± 1.69	12.20bc ± 1.69	15.89b ± 1.69	8.57c ± 1.69	8.57c ± 1.69	11.77bc ± 1.69	9.28c ± 1.69	9.82bc ± 1.69	11.72bc ± 1.69
K^+^	6.60b ± 0.67	6.53b ± 0.67	6.03b ± 0.67	10.97d ± 0.67	11.27cd ± 0.67	11.40bcd ± 0.67	12.97abcd ± 0.67	12.97abcd ± 0.67	13.40abcd ± 0.67	13.47abc ± 0.67	13.77abc ± 0.67	13.90a ± 0.67
**OM (%)**	0.51d ± 0.01	0.51d ± 0.01	0.50d ± 0.01	0.80c ± 0.01	0.79c ± 0.01	0.78c ± 0.01	0.85b ± 0.01	0.85b ± 0.01	0.83b ± 0.01	0.90a ± 0.01	0.89a ± 0.01	0.88a ± 0.01
**TOC(%)**	0.30d ± 0.01	0.29d ± 0.01	0.29d ± 0.01	0.46c ± 0.01	0.46c ± 0.01	0.46c ± 0.01	0.49b ± 0.01	0.49b ± 0.01	0.48b ± 0.01	0.52a ± 0.01	0.52a ± 0.01	0.51a ± 0.01
**Saturation(%)**	34.19c ± 0.25	0.028d ± 0.25	34.53c ± 0.25	37.06e ± 0.25	36.67e ± 0.25	36.37e ± 0.25	43.32bcd ± 0.25	43.32bcd ± 0.25	42.69d ± 0.25	44.32a ± 0.25	43.88ab ± 0.25	43.69abc ± 0.25

*Mean value (n = 3) ± Standard error

Different alphabetical letters showed significant (P ≤ 0.05) difference among treatments and vice versa

Sp. 1 *= Eucalyptus camaldulensis*, Sp. 2 *= Vachellia nilotica*, Sp. 3 *= Dalbergia sissoo*

## 4. Discussion

The results of current study revealed that minimum growth was found in the plants of control treatment. Salinity negatively affected plants growth because in saline soils, Na+ and Mg2+ can replace K [13]. This replacement affects the biochemical processes, protein synthesis, photosynthetic rate, and chlorophyll production in plants [12]. In addition to that, cell morphology and stomatal conductance are negatively affected due to salinity, which ultimately may lead to yield reduction and/or plant mortality [11, 49, 50].

*Eucalyptus camaldulensis* and *Vachellia nilotica* showed the ability to grow in salt affected soils because trees can minimize salt deposition and salt accumulation in the upper layer and surface layer of soil, respectively [51, 52]. Trees facilitate the leaching of salts by improving water permeability, and they tend to reduce electrical conductivity (EC), pH, and exchangeable sodium percentage (ESP) of soils [8, 53].

All rates of biochar application have shown very positive results in reducing the toxicity of sodium ions in saline soils. First of all, it reduced uptake of sodium ion (Na^+^) and enhanced uptake of potassium ion (K^+^), thus making sodium ions less available for plants and reducing its toxic effect [25, 54–56]. Furthermore, biochar application directly influenced processes of Na^+1^ leaching, sodium adsorption ratio (SAR), and electrical conductivity (EC) [56, 57] (Wang et al., 2020; Zhang et al., 2020). Biochar showed the tremendous ability to speed up the leaching process of salts that enhanced plant growth [58–60].

The results of current study revealed that the use of biochar enhanced plant growth to a certain extent, but the use of biochar in excessive amounts was not helpful as it deteriorated plant’s health. The use of biochar at the rate of 3% (w/w) increased morpho-physiological characteristics of selected tree species to some extent. It here was maximum increased when biochar was used at the rate of 6% (w/w). Still, when the biochar application rate was increased up to 9%, the growth and other physiological characteristics of plants started to deteriorate. So, appropriate use of biochar level is very necessary to grow plants in salt-affected soils. Our results are in accordance with previous studies as it has been reported that when biochar was applied at higher rates, it increased sodicity. The increase in sodicity resulted in decline in growth [61]. Other researchers have also reported that the application rate of biochar is an important component to determine the effectiveness of biochar [62, 63].

In another study, effects of different rates of biochar 0, 2, 4, and 8% (w/w) were determined on the growth of sorghum (*Sorghum bicolor L*.) seedlings under saline conditions, and it was reported that biochar application at a higher rate of 8% (w/w) had a negative influence on seedlings growth. The application of BC amendment showed the ability to decrease antioxidant enzymatic activities of CAT, POD, and SOD under salinity stress but higher application rate of biochar 8% (w/w) showed no significant impact on antioxidant enzyme activity [64]. In another study, a higher application rate of wheat straw biochar resulted in decreased growth of faba beans under saline conditions. The application rate of biochar was suggested at 2.5% (w/w) instead of 3.75% (w/w) because higher application rate of biochar resulted in increased salinity [65]. Coniferous wood biochar was applied at different rates 0%, 25%, 50%, or 75% (by volume) in the growing substance (peat-based) to check its effect on the growth and ornamental quality of two Lavender species (*Lavandula angustifolia* and *L*. *dentata*). It was reported that higher application negatively affected plant growth and physiological characteristics and also deteriorated soil qualities by increasing pH and EC of soil. Moreover enhanced rate of biochar application resulted in decrease of water retention capacity and nutrient availability [66].

Chlorophyll contents of plants were also decreased by applying biochar at higher rates. Our results are in accordance with previous studies as it has been reported that a higher application rate of wood biochar resulted in reducing the SPAD values of basil and tomato plants after obtaining maximum growth at optimum levels of biochar [67]. The growth of petunia plants was also decreased at higher rates of biochar application [68]. Leaf chlorophyll contents and photosynthetic rate of *Rosa rugose* plants were decreased by increasing the biochar percentage in growing substrates which is similar to the findings of this research [66].

Biochar was applied at the rate 0, 1.0%, 2.0%, 2.5%, 5.0%, and 10.0% (w/w) to check its effect on the growth of *Miscanthus lutarioriparius* in coastal saline-alkali soils. This study suggested that biochar was more beneficial at the application rate of 2.0% and 2.5% compared to 5.0%, and 10.0% (w/w), which is in accordance with our findings [69]. The electrical conductivity of soils treated with 9% (w/w) biochar was more as compared to 6% (w/w). Other studies also reported that excessive biochar is responsible for causing problems like increasing salinity instead of remediating the problems [70]. So, an appropriate level of biochar to remediate saline soil is very necessary.

In the current study, the biomass of three different species increased when biochar was applied from 0 to 6% (w/w). It was reported that as the rate of biochar application was increased from 0 to 5 kg/m^-2^, the dry biomass yield of four different types of vegetables increased up to 350% [71]. Biochar was applied at different rates (0, 10, 50, and 120 t ha^−1^) to check its effect on growth and biological nitrogen fixation rates. The results of the study showed that maximum biomass was obtained when biochar was applied at 10 t ha^-1^. According to the current study’s findings, as the rate of biochar application was increased to 120 t ha^-1^, biomass production of red clover was decreased significantly. [63].

Wood-derived biochar prepared at 350°C and 800°C was applied at four different rates of application 0, 1, 2, and 4% w/w to check its effect on corn crops. Results indicated that higher application rates resulted in crop growth and increased soil pH [72]. Another study reported that the application rate of biochar significantly affected greenhouse gas emissions in subtropical plantations. Biochar was applied at the rate of 0, 2, 5 and 10 t ha^-1^ and relationship between different gases was significantly different according to the application rate of biochar [73].

Biochar prepared from jarrah and pinewood was applied at different rates to check its effect on nitrogen cycling and wheat biomass. It was reported that the application rate of biochar higher than 29 t ha^-1^ resulted in a 39% reduction in grain biomass and growth of wheat [74]. Straw biochar was applied at six different rates 0%, 1%, 3%, 5%, 15% and 30% (w/w) to study its effect on the growth of maize plants. Results indicated that morphological characters (stem diameter, plant height, and root length) and physiological characters (chlorophyll contents and photosynthetic increased by 1 to 5% and then started to decrease up to 30% application rate [75]. A higher application rate (5% w/w) of wood biochar prepared by *Gliricidia sepium* was reported to deteriorate soil enzymatic activities as compared to lower application rates (1% and 2.5% w/w) [76].

Lettuce showed better growth when treated with cherry wood biochar at a 2% (w/w) application rate as compared to 3% (w/w) [77]. The combined effect of biochar and nitrogen fertilizers was tested on the growth of maize plants in alkaline soils. It was reported that 1% (w/w) biochar combined with 50% (of recommended dose) of nitrogen showed optimum results as compared to 2% (w/w) biochar combined with 100% (of recommended dose) of nitrogen [78]. Wine leese derived biochar was applied at different rates. Results of the study indicated that a higher biochar application rate (2% w/w) enhances the fertility of the soil. In contrast, the highest plant growth, enzymatic and bacterial activity was found when biochar was applied at the rate of 1% (w/w) [79].

Wheat straw biochar was applied at four different rates and 0.5%, 1%, 2%, and 4% by weight to coastal saline soil, and results showed that biochar at the application rate of 0.5% and 1% were more helpful in retaining soil nitrogen as compared to 2% and 4% [14]. Four different types of biochar were applied at three different rates 10 t ha^-1^, 20 t ha^-1,^ and 40 t ha^-1^ on the growth of *Lolium perenne*, and 10 t ha^-1^ was found to be most effective for plants growth and improvement of soil physicochemical characteristics [80].

Biochar was very effective in mitigating the negative effects of cadmium contaminated saline soil and enhanced all physiological and morphological parameters of wheat, but at higher biochar application rates, it showed negative effects [47]. Biomass and growth of cucumber are reported to decrease when sewage sludge was applied at higher rates 50g kg^-1^ than 10, 20, 30, and 40 g kg^-1^ [81]. Biochar was applied at the rate of 0, 5, 10, 20, 30, 40, and 50 (t ha^-1^) to check its effect on the growth of wheat grown under saline conditions. Grain yield of wheat was increased by 2.9% to 19.1% when biochar was applied at the rate of 5–10 (t ha^-1^) and when the rate of biochar was increased, it negatively affected the grain yield of wheat [82].

Biochar amendment applied at four different (0, 2, 4, and 8% by mass of soil) was reported to increase yield, photosynthetic rate, and stomatal conductance of tomato plant under saline water irrigation. Different application rates affected differently for morpho-physiological parameters of plants [83]. Lower rates of gypsum and biochar are reported to be more efficient in reducing nitrogen losses from coastal saline soil [84].

Higher amount of biochar decreased plant growth which may be due to the following reasons. Excessive amount of biochar results in increased salinity [65]. Higher application rate of biochar can also increase sodicity of soil [61]. Moreover it can also deteriorate soil health conditions by increasing the values of EC and pH [66]. Higher amount of biochar can decrease the leaf chlorophyll contents and photosynthetic rate of plants [66, 67]. Soil enzymatic activities are also deteriorated by excessive use of biochar [76]. Higher amount of biochar shows no significant impact on antioxidant enzymatic activities [64]. Moreover water holding capacity and nutrients retention capacity of soils is also deteriorated by the use of excessive amounts of biochar [66]. So, while using any type of biochar for remediation purposes, it is necessary to quantify the optimum level of biochar.

## 5. Conclusion

Salinity is the global issue; however, it is severe in the regions having arid climate and dependent on irrigational water for agriculture like Pakistan. Afforestation of salt affected soils is the conventional approach being used for their reclamation and amelioration, but growth plants is highly affected due to higher level of salts. It is observed that use of organic amendments can enhance plant growth and improve soil physicochemical characteristics of saline soils.

The current study results revealed that *Eucalyptus camaldulensis* is best tree species to grow in saline soils as compared to *Vachellia nilotica* and *Dalbergia sissoo*. *Eucalyptus camaldulensis* and *Vachellia nilotica* both showed promising result to remediate salt affected soils while *Dalbergia sissoo* showed poorest results. All levels of farmyard manure biochar showed better results as compared to control for all growth and physiological characteristics of plants. Among different levels of biochar, 6% (w/w) was found to be the best application rate as compared to 3% and 9%. Growth of all species increased with increasing the rate of biochar up to a certain extent and then started to decline. So, optimum level of biochar should be used to obtain maximum benefit for all selected tree species. Further research is needed to check the effect of different levels of biochar and survival of these plants in field conditions.
